# Deep Learning Enabled Diagnosis of Children's ADHD Based on the Big Data of Video Screen Long-Range EEG

This article has been retracted.

**DOI:** 10.1155/2022/5222136

**Published:** 2022-04-04

**Authors:** Dingfu Zhou, Zhihang Liao, Rong Chen

**Affiliations:** ^1^Department of Paediatrics, Huizhou Municipal Central People's Hospital, Huizhou, Guangdong 561000, China; ^2^Department of Electrophysiology, Huizhou No. 2 Maternal and Child Health Hospital, Huizhou, Guangdong 561000, China

## Abstract

Attention-deficit hyperactivity disorder (ADHD) is a common neurodevelopmental disorder in children. At the same time, ADHD is prone to coexist with other mental disorders, so the diagnosis of ADHD in children is very important. Electroencephalogram (EEG) is the sum of the electrical activity of local neurons recorded from the extracranial scalp or intracranial. At present, there are two main methods of long-range EEG monitoring commonly used in clinical practice: one is ambulatory EEG monitoring, and the other is long-range video EEG monitoring. The purpose of this study is to summarize the brain electrical activity and clinical characteristics of children with ADHD through the video long-range computer graphics data of children with ADHD and to explore the clinical significance of video long-range EEG in the diagnosis of children with ADHD. For a more effective analysis, this study further processed the video data of long-range computer graphics of children with ADHD and constructed several neural network algorithm models based on deep learning, mainly including fully connected neural network models and two-dimensional convolutional neural networks. Model and long- and short-term memory neural network model. By comparing the recognition effects of these several algorithms, find the appropriate recognition algorithm to improve the accuracy and then establish a recognition method for the diagnosis of children's ADHD based on deep learning long-range EEG big data. Finally, it is concluded that long-term video EEG can analyze the EEG relationship of children with ADHD and provide a diagnostic basis for the diagnosis of ADHD.

## 1. Introduction

ADHD is a common neurodevelopmental disorder in children and adolescents. Studies have found that the incidence of ADHD in American school-age children is not less than 4% [1]. A recent survey pointed out that the incidence of ADHD in school-age children is 5.9%–7.1%. Another retrospective study reported that the global incidence of children with ADHD was 5.29%–6.48% [2]. Studies have found that the incidence of ADHD in males and children is significantly higher than that of females [3–5]. Clinical studies have observed that the functional impairment of ADHD boys is equivalent to that of ADHD girls. At the same time, ADHD being prone to coexist with other mental disorders is one of its salient features [6], and it is necessary to pay attention to and treat these comorbidities in clinical treatment [7]. Comorbid mental disorders can affect the clinical manifestations and prognosis of children with ADHD [8], and in the long run, it will also reduce the individual's social adaptability in adulthood, such as increasing the rate of poor social relations and unemployment [9]. Understanding the incidence of ADHD, clarifying the differences in its distribution among different ages, genders, and clinical types, and further exploring the incidence and its influencing factors will help to better understand the clinical significance of each subtype of ADHD, and it may provide clues for exploring the etiology of comorbid diseases. Compared with Western countries, there is currently less attention and research on ADHD in Asia [10], and there are fewer relevant clinical studies and reports in China. In the process of prevention and treatment of ADHD, it is very important to accurately diagnose the disease. Its purpose is to properly handle the disease and enable the children to obtain and maintain a healthy and normal life. The best way to diagnose ADHD in children is through careful observation and recording of symptoms by medical staff and a comprehensive neurological examination. When conducting medical examinations on children, EEG examinations are usually indispensable. It uses a specific instrument to record the weak electrical signals generated by brain neurons collected by electrodes placed on the patient's head, and the amplified signal image EEG is often used to assist in the diagnosis of brain related diseases. ADHD can cause abnormal EEG curves, so the detection and diagnosis of ADHD is one of its most important applications. For medical staff, since the analysis of EEG and the judgment of ADHD are heavily dependent on professional physicians, the task of analyzing EEG alone is extremely heavy, and they are often faced with a large amount of complex data, in order to achieve monitoring. The accuracy of the EEG accumulated by each child ranges from ten hours to several days. It is very time-consuming to rely solely on manpower analysis, and the efficiency is very low. There are obvious differences in the characteristics of different children, and affected by the degree of professionalism, different medical staff may also get different results, which affects the accuracy of ADHD diagnosis. Therefore, in recent years, there have been more researches using computers as an auxiliary means of EEG analysis, and clinical applications have also become more and more. In the field of algorithms, more and more scholars have also applied deep learning and other theories to epileptic seizure detection, and various results have emerged one after another.

In this paper, we are going to summarize the brain electrical activity and clinical characteristics of children with ADHD through the video long-range computer graphics data of children with ADHD and to explore the clinical significance of video long-range EEG in the diagnosis of children with ADHD. For a more effective analysis, this study further processed the video data of long-range computer graphics of children with ADHD and constructed several neural network algorithm models based on deep learning, mainly including fully connected neural network models and two-dimensional convolutional neural networks model and long- and short-term memory neural network model. Main contributions of this paper are as follows:

- Utilize video long-range computer graphics data to conclude the brain electrical activity and clinical characteristics of children with ADHD
- Two-dimensional convolutional neural network model and long- and short-term memory neural network model were integrated
- By comparing the recognition effects of these several algorithms, find the appropriate recognition algorithm to improve the accuracy, and then establish a recognition method for the diagnosis of children's ADHD based on deep learning long-range EEG big data

The remaining paper is organized as follows:

In the subsequent section, a brief literature review of the most relevant and recent articles is presented which is followed by the detailed description of the design and development of the proposed methods. In Section 4, experimental results and observations of the proposed model in resolving the underlined issues are presented to verify its effectiveness. Finally, concluding remarks are given along with possible future directives.

## 2. Related Work

Research on the brain structure and function of ADHD patients has found that the function of some brain regions is inhibited, which has a negative impact on social interaction, academic achievement, and employment of ADHD patients. At the same time, other symptoms associated with ADHD, such as aggressive behavior, irritability, and ADHD comorbidities (opposing defiant disorder, conduct disorder, anxiety, and depression disorder), will also increase the above functional impairment [11]. The high incidence of ADHD and the comorbidity of behavioral problems need to arouse the attention and attention of clinicians, parents, and society. The etiology of ADHD is unclear. In the past, more researches focused on the development of functional brain areas and neurotransmitter changes. In the past five years, a series of advances have been made in the research on the etiology of ADHD, and the research results in biogenetics are particularly eye-catching. Heredity has an important influence on the pathogenesis, treatment, alleviation, and neurobiology of ADHD. Biederman *J* pointed out that if parents and siblings have a history of ADHD in the family, the risk of ADHD for this child will be 5–10 times higher than that of children in ordinary families [12]. Other studies have shown that the heritability of ADHD is about 70%–80% [13]. Bioinformatics studies have found the main symptoms of ADHD-attention deficit and hyperactivity/impulsiveness, there are more allelic regulatory genes, and there are independent related genes [14]. Epidemiological investigations found that the environmental factors related to ADHD include prenatal and childhood mothers and children's psychosocial dilemma, maternal mental factors, violence, stress, smoking, and drinking. Pires and his colleagues conducted a longitudinal study in Brazil: investigating the family environment of children with ADHD and their mothers' pregnancy and childbirth conditions, and reporting long-term follow-up behaviors of children based on the observations of the children's relatives (such as mothers). The study found that children with family dysfunction, mothers' lack of social support, adverse life events, and mothers with various family disagreements during pregnancy are at higher risk of being diagnosed with ADHD [15]. Another study found that children who experienced violence during prenatal and childhood, especially domestic violence, are more likely to suffer from ADHD [16]. The changes of brain structure and function in children with ADHD are diverse. A number of studies have found that as a special group of ADHD patients, brain volume is negatively correlated with ADHD symptoms [17]. Studies have found that due to the reduction of brain gray matter in ADHD patients, their brain volume is on average about 3%–5% less than that of healthy controls [18]. In addition, another study found that the volume of the right globus pallidus, right putamen, caudate nucleus, and cerebellum of ADHD patients' brains is smaller than that of normal people [19]. Another meta-analysis of MR diffusion tensor imaging research found that ADHD patients have extensive variations in the white matter of the brain, the frontal part of the corpus callosum radiation, the bilateral internal capsule, and the left cerebellum.

EEG is the sum of local neuron electrical activity recorded from extracranial scalp or intracranial. The waveform of EEG is composed of basic elements such as frequency, amplitude, phase, and waveform. The inspection of EEG is to analyze these basic elements and their interrelationships and further analyze their characteristics in time series and spatial distribution [20]. Since the 1920s, brain electrical activity can be recorded from the surface of the human brain; in the 1930s, people thought of monitoring the patient's EEG for a long time, but this was not possible due to technical problems; after the 1970s, with the development of electronic technology and computers, long-term EEG monitoring has become possible; after entering the 1980s, the rapid development of computer technology led to the rapid development of long-range EEG, and now EEG monitoring has reached the full level of digital video EEG. At present, there are two main methods of long-range EEG monitoring commonly used in clinical practice: one is ambulatory EEG monitoring, and the other is long-range video EEG monitoring (VEEG). The advantages of VEEG are as follows. (1) Observe the patient's clinical seizures through video recording, while simultaneously observing the patient's brain electrical activity before, during, and after the seizure, so as to more accurately judge the patient's seizure nature and seizure type. (2) The synchronization of EEG monitoring and video can help eliminate various interference artifacts, thereby reducing the rate of misdiagnosis. Disadvantages of VEEG are as follows. (1) The wired cable is connected to the EEG host, which limits the patient's activities, and children often cannot tolerate long-term monitoring. (2) The scope of camera monitoring is limited, and sometimes it is impossible to accurately capture all clinical manifestations of patients. (3) The patient must be hospitalized to complete the monitoring, which sometimes affects the patient's normal sleep cycle and seizure pattern.

Deep learning (DL) is a very important branch in the field of machine learning (ML), which is inextricably linked to machine learning. It is generally believed that the research of machine learning began in the 1950s. After years of development, machine learning has become a new type of multifield interdisciplinary, involving probability theory, statistics, approximation theory, biology, neurophysiology, and other fields. Computer science is a science that studies how to use computers to simulate or realize human brain learning activities. It is one of the most cutting-edge researches in the field of artificial intelligence. The research content of traditional machine learning mainly includes decision trees, artificial neural networks, support vector machines, K nearest neighbors, Bayesian classification, random forests, logistic regression, and other directions. The concept of deep learning comes from the artificial neural network in machine learning. It is based on a multilayer artificial neural network. It combines the low-level features of the data to form a more abstract, high-level feature that can represent the data attribute category and achieve efficient and automatic integration and extraction of its hidden features and inherent law information in large-scale data. Artificial neural network (ANN) is a mathematical model based on the theory of network topology and imitating the structure of the human central nervous system, especially the brain, as well as its complex information processing mechanism. It is used to perform operations on the input data. The 1940s was the beginning of neural network research. In 1943, American psychologist Warren McCulloch and mathematician Walter Pitts jointly published a paper [21], which proposed the MP model, which directly imitated human neurons the structure and working principle of the MP model are extremely simple, but it lays the foundation for later generations to study the neural network model. When researchers use machine learning algorithms to classify signals, they need to manually extract multiple features of the signal. The quality of the output of the algorithm depends heavily on the quality of the input signal features. Therefore, researchers need to accumulate a lot of experience and spend a lot of energy to explore and select features in order to improve the accuracy of the algorithm.

## 3. Proposed Methodology

### 3.1. Data Collection and Processing

#### 3.1.1. Data Collection

The experimental data obtained in this study are all from the newly diagnosed children of 6–16 years old who were diagnosed with ADHD in a children's hospital, and they have not been evaluated and treated for ADHD in the past. All patients used the CADWELL video EEG monitoring system in the United States. According to the international 10/20 system electrode placement standards, the electrodes filled with conductive paste were fixed with tape to the corresponding positions, and the monitoring time was at least 24 hours. The judgment of the long-range EEG on the screen is to compare the EEG of the patient, record the difference value of various waves, and then process it.

#### 3.1.2. Data Processing

Data standardization processing is as follows. The dataset studied in this article has only one type, that is, the brain wave difference value. However, during the data collection experiment, we found that the brain wave difference value of each of these ADHD child volunteers has different distribution ranges, so in the research of this article, data standardization is indispensable. There are many types of data standardization methods, the most typical of which is the normalization of the data; that is, the data is uniformly mapped to the (0, 1) interval. Commonly used are minimum-maximum normalization, zero-mean normalization, and other nonlinear normalizations.

The minimum-maximum standardization can directly scale the original data linearly to the interval (0, 1). The scaling function is

(1) $$\begin{array}{c} x^{*}=\frac{x-\min}{\max-\min}, \end{array}$$

where *x*^*∗*^ is the normalized value, *x* is the original value, min is the minimum value of sample data, and max is the maximum value of sample data.

Since the difference value sample data collected in this experiment is positive and negative, it represents the direction information of the difference value data along the coordinate axis. In order to retain this important data feature, the data standardization process in this article does not directly use the minimum and maximum standardization method. But to modify the method so that it can linearly scale the original data to the (−1, 1) interval so as to retain the direction information, the new formula is

(2) $$\begin{array}{c} x^{*}=\frac{2x-\left(\min-\max\right)}{\max-\min}. \end{array}$$

After a series of sorting and analysis of the collected raw data, we have obtained a dataset that is very suitable for the study of the neural network model based on deep learning.

### 3.2. Fully Connected Neural Network

#### 3.2.1. Basic Principles

Simulating the structure of human brain neurons in their paper, although the neural network has developed into a rather complex modern theory of multidisciplinary integration, various neural networks with different structures, characteristics, and functions are emerging in an endless stream, but their most basic components are still unchanged, and the McCulloch–Pitts neuron model is still used today.

The McCulloch–Pitts neuron model abstracts the above process into a mathematical model. In the artificial neural network model, artificial neurons become its basic structural unit, and they play the functions of receiving input data, processing data, and outputting data. When a neuron receives data from *n* other neurons connected to it, the neuron structure will associate *n* input weights, namely, *ω*_1_*ω*_2_*ω*_3_ … *ω*_*n*_ and these *n* input data. Multiply and calculate their weighted sum and then compare this weighted sum with its own threshold *b* and finally input the result of this comparison into the activation function *f* for calculation to obtain the output *y* of the neuron model. The formula is as follows:

(3) $$\begin{array}{c} y=f\left(\sum_{i=1}^{n}\left(x_{i}w_{i}-b\right)\right), \end{array}$$

where *x*_*i*_ is the input data of the *i* neuron, *w*_*i*_ is the connection weight of the *i* neuron, *b* is the threshold of this neuron, *f* is the activation function, and *y* is the output data of this neuron.

In the neuron model, the existence of the activation function is to realize the nonlinearity of the deep neural network. If the output of each neuron structure is multiplied by a nonlinear function, then the entire deep neural network will become a nonlinear model. In this way, the deep neural network we construct can theoretically approximate any function. This nonlinear function is what we call the activation function. There are three commonly used nonlinear activation functions, namely, tanh function (hyperbolic tangent function), sigmoid function, and ReLu function. The formulas of these three functions are

(4) $$\begin{array}{c} f_{\text{Relu}}\left(x\right)=\max\left(x,0\right),\\ f_{\text{sigmoid}}\left(x\right)=\frac{1}{1+e^{-x}},\\ f_{\tanh}\left(x\right)=\frac{1-e^{-2x}}{1+e^{-2x}}. \end{array}$$

Each of the above three activation functions has its own advantages. Sigmoid is a commonly used nonlinear activation function before. It can map the continuous value of the input to the interval (0, 1), and the tanh function can map the real number of the input to (−1, 1) in the interval.

#### 3.2.2. Optimization Algorithm

For the optimization of the loss function, the ADHD diagnosis problem studied in this paper is a typical two-classification problem in the supervised learning method. The problem of classification needing to be solved is how to accurately classify different sample data into preset categories. When there are only two categories, it is called a binary classification problem. In the classification problem, cross entropy is a very commonly used loss function; it can well describe the distance between two probability distributions, that is, the classification result output by the neural network and the actual classification of the sample data distance. The problem studied in this paper is a two-class situation, so the final result of the neural network model needs to be predicted. There are only two cases when the neural network predicts a sample: the sample belongs to the first category (i.e., the positive sample, in this article). In the research, the probability of children with ADHD is *p*, the probability that the sample belongs to category 0 (negative samples, normal children) is 1-p, and the true attribute of the sample is *y* (y for positive samples is 1 and for negative samples when *y* is 0); the cross entropy can be expressed as follows:

(5) $$\begin{array}{c} L=\frac{1}{N}\sum_{i=1}^{N}-\left[y_{i}\log\left(p_{i}\right)+\left(1-y_{i}\right)\log\left(1-p_{i}\right)\right], \end{array}$$

where  *y*_*i*_ is the attribute of *i* sample, positive sample is 1, negative sample is 0, *p*_*i*_ is the probability that *i* sample belongs to positive sample, and *N* is the number of samples.

However, since the output of neural network is not necessarily a probability distribution, we cannot directly regard the output of the model as probability P and apply it to the formula of cross entropy. Therefore, we need to convert the output results of the model into probability distribution, and softmax regression method is adopted in this paper.

Softmax regression can map the output value of the neural network to the interval of (0, 1), and the values after the mapping add up to 1, satisfying the nature of the probability distribution, so we can take these values after softmax regression processing is the probability, which is applied to the cross-entropy loss function. For this study, assuming that the original output of the neural network is *y*1 and *y*2, then the output after softmax regression processing is as follows:

(6) $$\begin{array}{c} \text{softmax}{\left(y\right)}_{i}=y_{i}^{\prime }=\frac{e^{y_{i}}}{e^{y_{i}}+e^{y_{2}}}. \end{array}$$

It can be seen that the new output meets all the requirements of the probability distribution, so this new output can be understood as the derivation of the neural network model. What is the probability that a certain sample is in these categories, so that the cross-entropy loss function can be used to determine calculate the distance between the probability distribution predicted by the model and the probability distribution of the true attributes of the sample.

#### 3.2.3. Model Construction and Training

Combining the neuron models described above according to a certain level, a fully connected neural network is obtained. The model is shown in Figure 1.

It consists of input layer, hidden layer, original output layer, softmax regression layer, and final output layer. After the sample data is processed by the short-time Fourier transform, each piece of data contains 8 ∗ 9 or 72 data points. Therefore, the number of nodes in the input layer of the neural network is 72, and the hidden layer has 5 layers, each with 512.256, 256, 128, and 64 nodes, and all add ReLU activation function and dropout layer; the dropout rate is uniformly 0.5, because this article is studying the two-classification problem, so the output layer is 2 nodes, and the last layer is softmax regression layer.

### 3.3. Convolutional Neural Network

#### 3.3.1. Basic Principles

Convolutional neural networks (CNN) is a very popular neural network structure in the field of deep learning, named for its mathematical operation of convolution. The biggest feature of the convolutional neural network is its parameter sharing feature. Due to this feature, the convolutional network can reduce a lot of parameters than the fully connected network, reducing the complexity of the network model and accelerating the training speed of the model. The main structure of a convolutional neural network is a convolutional layer and a pooling layer.

#### 3.3.2. Convolutional Layer

The convolutional layer is the most important network layer in the convolutional neural network, and it is also the source of the name of the convolutional neural network. The function of the convolutional layer is to perform feature extraction on the input data, and the specific implementation of the feature extraction function is completed by the multiple convolution kernels (also called filters) contained in it. The convolution kernel is actually a small numerical matrix, which can continuously slide on the input data of the current network layer. Each time it slides, it performs a convolution operation with the current data, adds the results of these convolution calculations to the corresponding, then inputs the parameters of the bias term into the activation function, and arranges the obtained results in the order of the convolution kernel sliding, so that the input of the next layer of neural network is obtained, and the feature extraction of the current layer of data is completed. The convolution kernel is equivalent to the neuron structure of a fully connected neural network. It also contains similar parameters, weights, and biases to the neuron. The above-mentioned numerical matrix for convolution calculation with the input data is this convolution kernel unit the weight parameter of, the offset term added to the result of the convolution operation is the offset parameter of this convolution kernel unit. The specific convolution process is as follows:

(7) $$\begin{array}{c} g\left(i\right)=f\left(\sum x_{i}w_{i}+b_{i}\right), \end{array}$$

where *g*(*i*) is the convolution output data of the current node, *f* is the activation function, *x*_*i*_ is the input data of the current node, *w*_*i*_ is the weight parameter of the convolution kernel, and *b*_*i*_ is the bias parameter of the convolution kernel.

The pooling layer is usually located between two convolutional layers. Its function is similar to that of the convolutional layer. It also extracts features from the input data. The pooling layer also has its own convolution kernel. Here, we call it a filter. The forward propagation of the pooling layer is completed by sliding the filter on the input data and performing calculations. However, the calculation of the pooling layer is no longer the weighted sum of the data and the weight is obtained, but a simpler method is adopted. In practice, the maximum value is commonly used, which we call the maximum pooling layer. Using the pooling layer can effectively reduce the size of the input data, so as to achieve the purpose of compressing the data and reducing the data dimension, which can effectively reduce the parameters in the network model, reduce the complexity of the model, and prevent the occurrence of overfitting.

#### 3.3.3. Model Construction and Training

Taking the classic LeNet-5 model as a reference, this paper constructs a convolutional neural network with one input layer, two convolutional layers, two pooling layers, two fully connected layers, and a softmax layer structure, as shown in Figure 2.

## 4. Experiments and Results

In this paper, all brain wave difference samples and normal samples of children with ADHD are mixed together and randomly shuffled to form a total dataset, and then the total dataset is divided into training dataset, test dataset, and verification data according to the practice of deep learning. Set three parts; each part accounted for 65%, 25%, and 10% of the total data. Among them, the training dataset is used for the model to fit the data features, that is, to optimize the parameters such as the weight and bias of the neural network. The validation dataset is used to verify the effect of the model after several rounds of training, so as to observe the effect of model training in real time, to find problems in model training in time, and to readjust the parameters of the model. The test dataset is used to evaluate the optimal model obtained after training and to measure the generalization ability and classification ability of this model.

### 4.1. Fully Connected Neural Network Training Results

The specific structural parameters of the fully connected neural network are shown in Table 1.

Likewise, the proposed model is trained using the combined data of all volunteers in the above-mentioned way. The TensorBoard visualization tool that comes with the TensorFlow framework is used to observe the entire training process in real time. During the training process, the model's recognition accuracy curve and loss value curve on the training dataset are shown in Figures 3 and 4.

As can be seen from the above figure, the recognition accuracy of the model is constantly increasing during the training process, and the loss value is constantly decreasing, indicating that the training process of the model is relatively stable, and there is no gradient explosion. During the training process, the model is training the accuracy rate on the set stabilized at about 94.5%, and the highest reached 96.5%. The recognition effect of the model on the training set is relatively good, and the effect on the validation set is slightly inferior, but it does not show much difference, indicating that the model has strong generalization ability and there is no overfitting.

### 4.2. Convolutional Neural Network Training Results

The dataset used for convolutional neural network training is still the combined dataset of all the volunteer children described above. The accuracy curve and loss value curve of the model on the training dataset during the training process are shown in Figures 5 and 6.

In the training process of this convolutional neural network, the accuracy of the model on the training set was stabilized at about 96%, and the highest was 99%. At the same time, the accuracy of the model on the validation set was stabilized at about 94.5%; the highest achieved 96%. Obviously, the convolutional neural network model has a very good recognition effect for ADHD diagnosis. Its recognition accuracy on the training set even reaches 99%, which means that it recognizes almost all states of the training set samples.

### 4.3. Model Testing and Comparison

Fully connected neural network is as follows. First, use the test set from the combined data of all volunteer children to test two fully connected neural network models that have completed training and obtained the best verification set recognition rate, and then use a separate test set of 5 volunteers. Independent tests were conducted on the two to observe the generalization ability of the model. The specific test results of the fully connected neural network model are shown in Table 2. It can be seen that the generalization ability of fully connected neural networks is quite good.

#### 4.3.1. Convolutional Neural Network

The test process is the same as that of the fully connected neural network model. The specific test results of the convolutional neural network model are shown in Table 3. We can see that the convolutional neural network model has an excellent effect on the recognition of epileptic seizures. The average accuracy rate of the model on the test set sample data reached 97.7%, and the average false negative rate dropped to 2.2%. This shows that the convolutional neural network model has a very strong generalization ability and can be used for the test set sample data of each volunteer the state you are in makes a very accurate identification and judgment.

Comparison of test experiment results is as follows. In this paper, we have tested the recognition effect of 2 kinds of 4 best deep learning models that were trained. Not only did we get the average recognition result of each model on the sample data of the mixed test set of all volunteer children, but also the average diagnostic effect of each model on the sample data of a single volunteer child test set is obtained. Compare the average evaluation indicators of these two neural network models. See Figure 7.

## 5. Conclusion and Future Directions

ADHD has brought great suffering to children, their families, and society. Therefore, research on the prevention and treatment of ADHD is of great positive significance. In the prevention and treatment of ADHD, early detection, early treatment, and early rescue are very important. The earlier the detection is, the earlier the child can receive drug treatment, thereby reducing the permanent nerve damage and mental torture caused by ADHD. It is necessary to make a diagnosis of ADHD in children as soon as possible and as easily as possible. In this paper, by analyzing the long-range EEG data of children with ADHD, two ADHD diagnosis methods based on deep learning are proposed, and the effects of these two recognition methods are tested and verified. The result is as follows. The ADHD diagnosis method of data preprocessing and deep learning model analysis proposed in this paper is very feasible. Generally speaking, the use of brain electrical signal data to classify and recognize ADHD diagnosis is the most accurate. However, the recognition method proposed in this article also has a good recognition accuracy for the brain wave difference data of children with ADHD. Especially for the convolutional neural network, its various indicators are basically the same as the recognition indicators of many deep learning classification methods based on EEG signals in the same period. This is of great significance for the long-range computer graphics of the video screen as the diagnosis basis for ADHD.

In future, we have planned to extend the operational capabilities of the proposed deep learning based model to other diseases as well.

## Figures and Tables

**Figure 1:** Fully connected neural network model.

**Figure 2:** Convolutional neural network model.

**Figure 3:** Training accuracy curve of fully connected neural network.

**Figure 4:** Training loss curve of fully connected neural network.

**Figure 5:** Convolutional neural network training accuracy curve.

**Figure 6:** Convolutional neural network training loss curve.

**Figure 7:** Comparison of the average evaluation indicators of the two models.

**Table 1:** Some structural parameters.

Parameter	Value
Initial learning rate	0.0012
Attenuation rate	0.95
Training batch size	20
Number of iterations	1000

**Table 2:** Specific test results of the fully connected neural network model.

Volunteer child number	Mean accuracy (%)	Mean underreporting rate (%)
1	96.5	1.2
2	90.8	3.5
3	94.5	4.3
4	93.2	8.9
5	90.1	7.6
Average value	92.7	5.1

**Table 3:** Specific test results of the convolutional neural network model.

Volunteer child number	Mean accuracy (%)	Mean underreporting rate (%)
1	96.5	2.3
2	97.4	3.5
3	98.6	1.7
4	99.3	3.1
5	96.4	2.6
Average value	97.7	2.2

## Data Availability

The datasets used during the current study are available from the corresponding author on reasonable request.
